# A Medical Image Fusion Method Based on SIFT and Deep Convolutional Neural Network in the SIST Domain

**DOI:** 10.1155/2021/9958017

**Published:** 2021-04-21

**Authors:** Lei Wang, Chunhong Chang, Zhouqi Liu, Jin Huang, Cong Liu, Chunxiang Liu

**Affiliations:** ^1^School of Computer Science and Technology, Shandong University of Technology, Zibo 255000, China; ^2^Anhui Key Laboratory of Plant Resources and Plant Biology, Huaibei Normal University, Huaibei 235000, China

## Abstract

The traditional medical image fusion methods, such as the famous multi-scale decomposition-based methods, usually suffer from the bad sparse representations of the salient features and the low ability of the fusion rules to transfer the captured feature information. In order to deal with this problem, a medical image fusion method based on the scale invariant feature transformation (SIFT) descriptor and the deep convolutional neural network (CNN) in the shift-invariant shearlet transform (SIST) domain is proposed. Firstly, the images to be fused are decomposed into the high-pass and the low-pass coefficients. Then, the fusion of the high-pass components is implemented under the rule based on the pre-trained CNN model, which mainly consists of four steps: feature detection, initial segmentation, consistency verification, and the final fusion; the fusion of the low-pass subbands is based on the matching degree computed by the SIFT descriptor to capture the features of the low frequency components. Finally, the fusion results are obtained by inversion of the SIST. Taking the typical standard deviation, Q^AB/F^, entropy, and mutual information as the objective measurements, the experimental results demonstrate that the detailed information without artifacts and distortions can be well preserved by the proposed method, and better quantitative performance can be also obtained.

## 1. Introduction

The pathology information displayed by medical imaging of different modalities plays a key role in modern medical diagnosis. Unfortunately, it is difficult to synchronously get the full-information images by one imaging device at the same time due to their different imaging principles [1]. Therefore, doctors have to spend more time and energy to read the medical information they want from different devices. A common method to deal with this problem is to fuse the multi-modal images from the same location of the body into one image, which is called the medical image fusion and has been widely used in medical image analysis, precision radiotherapy surgery, and computer-aided medical diagnosis [2].

Nowadays, various medical image fusion methods have been proposed, all of which can be roughly classified into two categories: methods in the spatial domain and in the transformed domain. Different from the former directly using some algebraic operations or filtering, the latter methods, capturing more features in different scales and directions, are the research hotspot. Such scheme usually contains three steps: decomposition, combination, and reconstruction [3].

From the fusion procedure, it is clear that the fusion performance is highly determined by the decomposition tools and the fusion rules. The tools play the role of providing the sparse representations of the features and the fusion rules play the role of transferring the features into the final fusion results. For the decomposition tools, the Laplace Pyramid transform cannot provide directional information; the typical wavelet transform only can decompose the images into three high-pass subbands in each level, so it is limited by the number of directions. The contourlet can get more directional subbands in each level, but the loss of shift-invariance is easy to result in the pseudo-Gibbs phenomenon [4]. For the fusion rules, the active level measurement-based rule [5] is popular; however, it is easy to produce the artifacts. Though some other fusion rules have been proposed, such as the SVM [6], PCA [7], ICA [8], etc., the fusion results are still unsatisfactory. It is important to consider the feature information during the implementation of the fusion rules [9]. Recently, there has been some good work to improve the fusion performance from these aspects. For example, in literature [10], it proposes a multi-modality image fusion method in the non-subsampled contourlet transform (NSCT), in which the high-pass subbands are integrated by the phase congruency-based rule and the low-pass subbands are combined by the local Laplacian energy-based rule. In literature [11], it proposes an image fusion framework, which integrates NSCT into sparse representation and a principal component analysis (PCA) is implemented in dictionary training to reduce the dimension of learned dictionary. The low- and high-pass coefficients are fused by the sparse representation and Sum Modified-Laplacian, respectively. In literature [12], the source multi-modality images are decomposed into cartoon and texture components. The cartoon components are combined by an energy-based fusion rule for morphological structure preservation and the texture components are combined by the dictionary training. In addition, some similar fusion schemes can be found in the literatures [13, 14]. Such schemes provide good fusion results for they have made full use the of the good mathematical properties of NSCT and the learning abilities of dictionary learning to capture the important features. The main disadvantage, however, is the time cost. The NSCT, the shift-invariance version of the contourlet transform, is too time-consuming because it has to use the non-subsampled band-pass filters to produce the shift-invariance. And the dictionary training usually suffers from the number and the dimension of the dictionary. It is easy to result in the dimensional disaster in the fusion.

Another research hotspot is the neural networks-based medical image fusion methods. Some good results have been reported, such as the artificial neural networks-based method, the Pulse Coupled Neural Network- (PCNN-) based method [15]. However, the fusion performance is limited by how to tune the parameters and the number of the layers in the traditional neural networks models. Very recently, the deep learning technologies, such as the deep convolutional neural network, have achieved great success in the areas of image classification and target recognition, as well as in image fusion. For example, literature [16] proposes a novel image fusion algorithm based on deep support value convolutional neural network, literature [17] proposes the medical image fusion with the all convolutional neural network, and literature [18] proposes a general image fusion framework based on convolutional neural network, which is called IF-CNN. Literatures [19, 20] review the recent advances and future prospects about deep learning for pixel-level image fusion. In the above methods, the good results are obtained for their better learning ability than the traditional neural network models. However, such methods are directly learned in the pixel level, losing the important feature information.

To deal with the above problems, a medical image fusion method based on the SIFT and CNN in the SIST domain is proposed. Different from other transformation tools, such as the wavelet and the contourlet, the SIST can decompose the images into high-pass and low-pass subbands to extract more useful features in different scales and directions. Besides, with the same shift-invariance as the NSCT, the calculation efficiency of SIST is higher. To make full use of the features in the source images, the fusion rule for the low-pass subbands is based on matching degree of the SIFT descriptor. The SIFT feature is based on the local points of interest on the object and is independent of the size and rotation of the image. So, its tolerance for changes in noise and micro-viewpoints is quite high [21]. From this point of view, it is more suitable than the structure features for medical image fusion. The fusion of the high-pass subband is based on the CNN-based scheme to employ the good learning ability of the CNN model.

The rest of the framework is organized as follows. The details of the proposed method are shown in Section 2. Experimental results with important discussions are shown in Section 3. Finally, the conclusion is shown in Section 4.

## 2. Methodology

The whole procedure of the proposed medical image fusion method is described in Figure 1. After the decomposition and directional partition in different scales, the coefficients of the source medical images are obtained. Then, the high-pass and low-pass coefficients of the fused image are produced by the corresponding fusion rules. Finally, the fusion results are obtained.

The principle of the proposed method can be specifically explained from three aspects to understand: firstly, from the tools of sparse representation in medical image fusion, the SIST has better mathematical properties to provide the good representations of the important features; secondly, the traditional fusion rules are easy to lose the captured feature information during the procedure of transferring them into the final results; thirdly, the transferred feature information is only in the low level and it is not abstract enough to do the feature fusion. Therefore, considering the above needs, a CNN model is pre-trained the get the deep and abstract features in the SIST domain and the SIFT-based fusion rule is developed.

### 2.1. The Shift-Invariance Shearlet Transform

The discretion of SIST mainly consists of two steps [21]: the multi-scale partition and the directional localization. To provide the shift-invariance, the former step is done by the non-sub-sampled pyramid filters, and the latter step is implemented by using the filters of shearing. Let *j* be the scale of image decomposition, *j*=1,2,…, *M*; the whole process can be summarized as the following steps.

(1) The image *f*^*j*^ is decomposed into low-pass image *f*^*j*+1^ and high-pass image *g*^*j*+1^ using the non-sub-sampled pyramid *f*.
(2) Construct the Meyer Window for the high-pass image *g*^*j*+1^:
    Generate shearing filter window *W* in pseudo-polarization grid;
    Map *W* from pseudo-polarized grid system to Cartesian coordinate system to generate a new shearing filter *W*_new_;
    Compute the 2*D* discrete Fast Fourier Transform (FFT) of *g*^*j*+1^ to generate the matrix *Fg*^*j*+1^;
    Apply band-pass filtering to the matrix *Fg*^*j*+1^ to compute different directional components.
(3) Directly re-assemble the Cartesian sampled values and apply the inversing 2-D FFT to produce the SIST coefficients.

The inversing transformation is the opposite process of the forward transformation. Since there is no need to use directional band-pass banks to get different directions like the NSCT; the SIST is more efficient. More details about the implementation can be found in literatures [22, 23].

### 2.2. The Fusion of the High-Pass Subbands

The procedure of the high-pass fusion is shown in Figure 2. Before the fusion, a CNN model is trained by the pre-fused images. The whole fusion process mainly consists of four steps: feature detection, initial segmentation, consistency verification [24–26], and the final fusion. In the first step, the high-pass subbands are input into the CNN model to output the score map, which contains the feature information of each high-pass subband. Each coefficient in the score map represents the feature attribute of a pair of corresponding blocks from two high-pass subbands. Then, by averaging the overlapping regions, a feature map of the same size is obtained from the score map. Furthermore, the feature map is segmented into a binary map with the threshold. In the third step, the consistency verification is implemented to refine the binary segmentation mapping to generate the decision map. Finally, the fused image is obtained by applying the pixel-weighted scheme on the decision map.

#### 2.2.1. Train the CNN Model

For a pair of medical image patches {*A, B*} of the pre-fuse images, the goal is to learn a CNN model whose output is a scalar ranging from 0 to 1. Specifically, when the feature is almost from *A* but not *B*, the output value should be close to 1, or the value should be close to 0. In other words, the output represents the feature degree of the pair of the image patches. Therefore, a large number of example pairs are used to be the training examples.

In Figure 3, the structure of the trained CNN model is shown. It has two identical architecture branches, each of which takes the medical image blocks as the input. According to [27], it is suitable to set the size of image block to 16 × 16. There are three convolution layers and a maximum pooling layer in each branch of the network. The size of neuron perception is determined by the core size of the convolution layer. In this paper, the core size is set to 3 × 3, the step size is set to 1, the scaling factor of the pooling layer is set to 2 × 2, and the span space is set to 2.

#### 2.2.2. The Feature Detection

Let *A*_*H*_ and *B*_*H*_ be the two high-pass subbands; a score map can be obtained once *A*_*H*_ and *B*_*H*_ are input into the constructed CNN model. The value of each coefficient in the score map ranges from 0 to 1, indicating the feature degree of a pair of 16 × 16 blocks. The closer that the value is to 1, the more concentrated patches are from image *A*_*H*_, and vice versa. In order to generate a feature map (represented as *M* here) of the same size, it assigns the value of each coefficient in the score map to all the coefficients of the corresponding block in *M* and averages the overlapping pixels.

#### 2.2.3. Initial Segmentation

In order to retain as much useful information as possible, the feature map needs to be applied on the maximum strategy. According to the experience, a *d* threshold of 0.5 is applied to the feature map to generate the binary map; that is, the focus map is divided by the following formula:

(1) $$\begin{array}{c} T\left(x,y\right)=\left\{\begin{array}{cc} 1, & M\left(x,y\right)>\tau ,\\ 0, & \text{otherwise,} \end{array}\right. \end{array}$$

where is *M* is the focus map, *T* is the binary map, is the *τ* threshold. According to our experience in the experiments, it is found that when the threshold equals 0.5, it is good enough for medical image fusion and it is suggested to be in the range from 0.4 to 0.7 for the other multi-modal image fusion.

#### 2.2.4. The Consistency Verification and Fusion

There may be some misclassified pixels in the above binary map, so it is necessary to remove these mistakes. The traditional method to deal with this problem is to use the threshold scheme, but it is easy to result in some unexpected artifacts around the boundary between the focused and defocused regions. Therefore, the guided filter [28], which is the effective edge-preserving filter to retain the structural information, is employed. There are two free parameters in the guided filtering algorithm: the local window radius *r* and the regularization parameter *ε*. In this paper, *r* is set to 8 and *ε* is set to 0.1. More details about its implementation can be found in [29]. Finally, the fused high-pass subbands can be obtained by the following weighted formula:

(2) $$\begin{array}{c} F_{H}\left(x,y\right)=D\left(x,y\right)A_{H}\left(x,y\right)+\left(1-D\left(x,y\right)\right)B_{H}\left(x,y\right), \end{array}$$

where *F*_H_ is the high-pass subband of the fused image, *D* is the decision map, and *A*_*H*_ and *B*_*H*_ are the corresponding high-pass subbands of the image to be fused, respectively.

### 2.3. The Fusion of the Low-Pass Subband

The fusion of the low-pass subband is based on the matching degree of the SIFT [29, 30]. Suppose fdesc_1_(*i*) and fdesc_2_(*j*) are the SIFT descriptor from the low-pass subbands of the two images to be fused, where *i* ∈ (1, *m*), *j* ∈ (1, *n*), and *m* and *n* are the total number of the SIFT descriptor, respectively. Then, compute the distance dist(*i*, *j*) between fdesc_1_(*i*) and fdesc_2_(*j*), and sort all the distances. Let 2nd BigDist(*i*, *j*) be the second largest value; if dist(*i*, *j*) < 2nd BigDist(*i*, *j*), the two SIFTs are called matched.

If fdesc_1_(*i*) and fdesc_2_(*j*) are matched, record their location, respectively. If the locations are also the same, it means that both of the content and the location of the region that computed the SIFT descriptors are the same [20]. Finally, the SIFT descriptors that meet the above conditions are recorded to generate a matching degree map match_map, where 1 < =*i* < =*n*. The low-pass subband of the fusion result can be obtained by the following formula:

(3) $$\begin{array}{c} F_{L}\left(x,y\right)=\text{match}\_\text{map}*A_{L}\left(x,y\right)∼\text{match}\_\mathrm{map*}B_{L}\left(x,y\right), \end{array}$$

where “∼” means the negation, *F*_*L*_ is the low-pass subband of the fused image, and *A*_*L*_ and *B*_*L*_ are the corresponding low-pass subbands of the image to be fused, respectively.

## 3. Results and Discussion

In this section, experiments in six groups are carefully done to show the performance of the proposed fusion method. Before the experiments, a CNN model is firstly trained under the public medical data set LIDC, Whole Brain Atlas, and the nature data set ImageNet. All the data sets are downloaded and pre-processed to be the same size of 256 × 256. To get the parameters of the CNN model, 2000 medical images from LIDC, 3000 nature images from the ImageNet, and 200 medical images from the Whole Brain Atlas are, respectively, used to produce the sub-model and the final model is integrated based on the three sub-models. The experimental platform is the INSPUR big data processing server NF5280M5, Intel Xeon CPU, 128 GB RAM.

Four famous medical image fusion methods, i.e. the Pulse Coupled Neural Network-based method (noted as PCNN) [31], the convolutional sparse representation based method (noted as CSR) [32], the Shearlet based method (noted as Shearlet) [33], and the Deep Convolutional Neural Network-based method (noted as DCNN) [34], are employed to prove the efficiency of the proposed fusion method (Proposed for short). All the parameters are set as the same as what they are reported in the corresponding literature. The decomposition level of SIST is set to 4 and the filters are all “maxflat.” After decomposition of each level, 32, 32, 16, and 16 high-pass subbands are obtained.

There is no gold standard for evaluating image fusion at present. The usual approach is to use subjectively visual comparisons and objectively quantitative comparisons. This convention is also followed in our paper. Standard deviation (SD for short), entropy (En for short), mutual information (MI for short), and *Q*^*AB/F*^ are used to be the objective evaluation measurements. SD measures the degree of single pixel value relative to the mean value. En shows how much information the image itself contains. MI shows how much information the fused image captured from the source images; *Q*^*AB/F*^ measures the edge information transferred from source image to fusion image. The greater the value of these measurements, the better the fusion results [35].

In Figure 4, the three groups in the first row are the gray CT and MRI images, and the three groups in the second row are the color CT and PET images from the patients of anaplastic astrocytoma and mild Alzheimer's disease, respectively. In each data set, the number of slices is 20, 15, and 21, respectively. To save the space, parts of the fusion results are shown in Figures 5 and 6, and the average of the objective evaluation is shown in Tables 1 and 2, respectively.

Though the information expressed by the above fusion images is better than the source image, the fusion results are different. By comparing the arrows of different colors in Figures 5 and 6, it shows that the edge of PCNN method is obviously blurred, and the individual character details (labeled by the blue arrows) and contour features (labeled by the yellow arrows) have been lost. For the Shearlet and DCNN method, the result is clear enough for its good learning ability, but the detail and texture are not good (labeled by the red and green arrows). The main reason is that it is directly learned in the pixel level. In contrast, the detail and texture structures in the fusion results obtained by the proposed method are much clearer, and the ghosting phenomenon can be effectively eliminated. It can be seen that the method proposed is better than CSR and Shearlet method in detail processing. Particularly, comparing the yellow arrow in Figure 6 for the DCNN and the proposed method, it obviously indicates that the information in the results obtained by the proposed method can be kept as what they are like in the source data. In addition, from the objective evaluation in Tables 1 and 2, it can be seen that the objective value of the proposed method is much higher than other methods under the four indicators, which further verifies that more feature information can be effectively captured and fully transferred into the fusion results by the proposed method, showing better visual sensing. All the results prove that more detail features from the source images can be captured and transformed well into the final results by the proposed method.

## 4. Conclusion

Based on the SIST and the CNN, this paper proposes a medical image fusion method, which makes full use of the multi-resolution and multi-directional characteristics of SIST, and also combines the self-learning advantages of CNN. According to the careful objective analysis and subjective comparison, experiments show that the target information and contour features can be well displayed in the final results. Besides, the artifacts and distortions can be effectively suppressed. Compared with other famous fusion methods such as the PCNN-based method, DCNN-based method, sparse representation-based method, etc., the proposed method can get better fusion results.

## Figures and Tables

**Figure 1:** The architecture of the proposed method.

**Figure 2:** The fusion procedure of the high-pass subbands.

**Figure 3:** The trained CNN model in this paper.

**Figure 4:** The six groups of source images. Every two of them are captured in the same location with different modalities,CT‐MRI in the first row and MRI‐PET in the second row.

**Figure 5:** The fusion results of the three groups of CT-MRI. (a) PCNN. (b) CSR. (c) Shearlet. (d) DCNN. (e) Proposed.

**Figure 6:** The fusion results of the three groups of MRI-PET. (a) PCNN. (b) CSR. (c) Shearlet. (d) DCNN. (e) Proposed.

**Table 1:** The objective evaluations of CT-MRI fusion in Figure 5.

Method	Group 1				Group 2				Group 3			
	SD	*Q* ^*AB/F*^	En	MI	SD	*Q* ^*AB/F*^	En	MI	SD	*Q* ^*AB/F*^	En	MI
PCNN	20.63	0.50	2.12	0.65	20.36	0.55	2.00	0.58	20.87	0.39	1.91	0.45
CSR	20.86	0.55	2.20	0.77	21.56	0.60	2.11	0.62	23.96	0.46	2.00	0.62
Shearlet	21.44	0.59	2.28	0.78	22.43	0.62	2.18	0.69	23.55	0.51	2.10	0.69
DCNN	22.35	0.71	2.31	0.82	23.58	0.68	2.26	0.76	24.20	0.55	2.19	0.78
Proposed	23.22	0.83	2.45	0.88	24.43	0.79	2.33	0.82	24.55	0.68	2.28	0.85

**Table 2:** The objective evaluations of MRI-PET fusion in Figure 6.

Method	Group 4				Group 5				Group 6			
	SD	*Q* ^*AB/F*^	En	MI	SD	*Q* ^*AB/F*^	En	MI	SD	*Q* ^*AB/F*^	En	MI
PCNN	35.62	0.59	3.76	0.46	41.05	0.62	4.11	0.38	31.12	0.58	3.89	0.62
CSR	37.21	0.65	3.88	0.50	43.56	0.72	4.25	0.42	33.93	0.65	3.96	0.71
Shearlet	37.64	0.67	4.13	0.59	44.95	0.78	4.35	0.48	34.52	0.69	4.31	0.76
DCNN	38.19	0.73	4.50	0.65	45.36	0.81	4.44	0.62	34.91	0.76	4.55	0.81
Proposed	39.42	0.84	4.65	0.70	47.21	0.86	4.63	0.63	35.68	0.83	4.87	0.85

## Data Availability

The data used to support the findings of this study are available from the corresponding author upon request.
